# Generative Adversarial Network for Musical Notation Recognition during Music Teaching

**DOI:** 10.1155/2022/8724688

**Published:** 2022-06-07

**Authors:** Na Li

**Affiliations:** School of Music and Performing Arts, Mianyang Teachers' College, Sichuan, Mianyang 621000, China

## Abstract

In order to improve the quality and efficiency of music teaching, we try to automate the teaching of music notation. With the addition of computer vision technology and note recognition algorithms, we improve the generative adversarial network to enhance the recognition accuracy and efficiency of music short scores. We adopt an embedded matching structure based on adversarial neural networks, starting from generators and discriminators, respectively, to unify generators and discriminators from the note input side. Each network layer is then laid out according to a cascade structure to preserve the different layers of note features in each convolutional layer. Residual blocks are then inserted in some network layers to break the symmetry of the network structure and enhance the ability of the adversarial network to acquire note features. To verify the efficiency of our method, we select monophonic spectrum, polyphonic spectrum, and miscellaneous spectrum datasets for validation. The experimental results demonstrate that our method has the best recognition accuracy in the monophonic spectrum and the miscellaneous spectrum, which is better than the machine learning method. In the recognition efficiency of note detail information, our method is more efficient in recognition and outperforms other deep learning methods.

## 1. Introduction

Computer simulations play a very important role in teaching music today. The greatest advantage of multimedia technology is cross-media presentation. The traditional school board is limited to written and face-to-face instruction, and much virtual knowledge cannot be displayed, so students cannot feel the main points of learning in a personal way. Thus, the development of computer technology today has made education presentable, and it can realize the conversion from text data to image video, also the conversion of music notation to audio, and also the virtual performance of musical instruments. The combination of computer technology and education has added more fun to education, and the novel teaching methods can mobilize students in all aspects, make the teaching mode more active, and improve the quality of teaching significantly.

The traditional model of music education is one-on-one teaching between teacher and student, and music-type art training is usually a small course. Lessons involving music notation are rather boring, and classroom-style instruction prevents students from getting a first-hand feel for the tones and distinctions of each musical notation. All music notation and musical notation require rote memorization by students to remember, which drastically reduces the quality of music notation instruction [1]. The advent of computer technology has improved the efficiency of teaching music notation [2]. With the aid of computer technology, various music software was born to bring great convenience to students' extracurricular music learning. Music software contains virtual instrument functions, digital score presentation functions, virtual arranging tools, and digital tuners. A series of music assistance programs have emerged to make self-learning music more convenient and are sought after by a large number of amateur music lovers [3].

Music notation initially existed in the form of handwriting, the construction of music scores in the early period of music festivals was based on the sense of sound, and the writing of all music symbols varied from person to person, which brought great challenges to the work of automatic music notation recognition. The fusion technology of computer vision and image recognition algorithm to realize the music score recognition can improve the working efficiency and save the working cost. To orderly carry out the music score recognition work and solve the problem of variation of handwritten scores, the researcher specially designed a notation frame, and each music notation frame can learn the handwriting habits of different musicians independently and will automatically label the information of music source, author, and genre after recognition [4–6]. The computer input work is performed by scanning the music notation manuscript, and each music symbol is designed in advance as a label for easy learning of the score. After the recognition is completed, musicians can download and edit the music from the Music Resource Sharing website.

Music notation recognition systems give more prominence to image recognition techniques, yet ignore the homogeneous heterogeneity of music notation handwriting. For this problem, the researchers used computer vision techniques for the same speciﬁcation. Each handwritten music notation has a different representation, and different types of music notation cannot be processed with the same heuristic [7]. According to the frequency of music notation usage, the scanned music notation needs to be reconstructed phonetically, and the music notation is assigned according to different weights as a way to cater to the fluency of the music notation. With the development of machine learning techniques, each note symbol in a musical notation can be generalized and model training can be achieved by manually building a note symbol dataset. So far, some researchers have demonstrated that the combination of note symbols and machine learning techniques is not suitable for all music notation, where note symbols captured by pentatonic scores need to be preprocessed with images to be applicable, and special music element classification requires dataset-independent production based on specific notes. Although the machine learning method is the first innovation in the research of music short score recognition, the method adds a lot of work cost to the method due to the lack of a clear and explicit engineering framework and the tedious manual labeling work, plus the accuracy and real-time performance of the machine learning method are not good enough. Therefore, there is still a lot of research space in the field of music score recognition [8, 9].

In the experiments of adversarial generative networks, we try to fuse music notation features into the generator to accomplish the task of music notation recognition by stimulating the generation of pseudo-samples. The musical notation recognition method we designed consists of symbol recognition and score reconstruction. The flowchart is shown in Figure 1. We adopt an embedded matching structure based on adversarial neural networks, starting from generators and discriminators, respectively, to unify generators and discriminators from the note input side. Then, each layer of the network is laid out according to the cascade structure, and then the residual blocks are inserted in some network layers to break the symmetry of the network structure and enhance the ability of the adversarial network to acquire note features. Finally, we validate the effectiveness of our method on a public dataset of music notation.

The rest of the paper is organized as follows.  Section 2 introduces the research history and research results of musical notation recognition.  Section 3 details the principles and implementation procedures related to the improved adversarial music notation recognition network.  Section 4 shows the experimental datasets and the analysis of the experimental results. Finally, Section 5 summarizes our research and reveals some further research work.

## 2. Related Work

There are many branches of music notation recognition research, among which optical music recognition is one of the well-known research branches. Optical music recognition mainly relies on optical factors to achieve the recognition of music symbols. The literature [10] has a very in-depth study on optical music recognition, and the authors try to establish a series of different stages to deal with the grading of music symbols. Considering the differences between low-order to high-order notes, the authors propose a general optical music recognition framework and supplement it with different note segmentation methods to achieve the task of nondifferentiated recognition of musical short scores. For special notes, the authors default to note segmentation for preprocessing and then unify all music symbols and treat them as independent phonemes for optical scanning.

Researchers in literature [11] tried to improve the recognition accuracy of music notation from the perspective of images, and they proposed a binarization algorithm, which can temporarily solve the problem of a small number of music notation images. However, the method lacks generalization, has limited applications, requires adaptation for note images with different characteristics, relies heavily on optical music recognition methods in the conversion between high and low order for different music scores, and becomes less applicable due to the lack of flexibility of a unified note recognition framework. Researchers in the literature [12–14], after validating a large number of machine learning methods, found that DNN models have a high degree of generalizability and are better at musical score recognition with better recognition accuracy. The application potential of deep learning methods in music short scores is high, but the method requires more stringent datasets. In the construction of the musical score dataset, the skewed manuscript content needs to be corrected in advance, and the overlapping notes need to be separated in advance according to the correct score. In addition, to improve the inclusiveness and increase the volume of the dataset, the literature [15, 16] proposed data enhancement algorithms to improve the coverage of different angles and sizes of note features in the dataset.

The study of musical notation is not a smooth process, in which music notation segmentation is a great challenge. Music notation is different from characters, which have a professional character library that can be used as a database to unfold the mapping. However, music symbols are a new task in the early stage of research, and without a huge music symbol library as data support, the music symbol database needs to be built from scratch, which undoubtedly brings great difficulties to the work of music score recognition. At the initial stage of music symbol database establishment, researchers chose to define the scanned documents of notes with poor image quality with small element labels and then separated the notes from pseudo-notes by noise threshold. Based on the former research method, the literature [17] proposed the principle of object reconstruction at the initial stage of notes, which solved the problem that the overlapping of notes and pseudo-notes at the initial stage of notes could not be separated. Considering that the workflow of the traditional note detection method is too tedious and the accuracy is low, the literature [18, 19] first tried to apply the region-based neural network method to note feature extraction, abandoning the note separation step, directly starting from note features, and training the model to directly complete note recognition. However, the method has high requirements on the dataset. Researchers in the literature [20] were again inspired by the musical notation baseline and used the baseline as the note criterion to build a variety of note and notation models to achieve excellent note recognition accuracy with an adaptive fusion approach.

To avoid differentiated conversions between higher and lower orders of notes, researchers in the literature [21, 22] chose a neural network approach that starts with the overall musical notation. They transformed the output of the neural network as a sequence of notes and then annotated the notes of higher and lower orders in the sequence position. The released note elements are converted to actual notes in backpropagation, preventing multiple repetitions of detection during postprocessing. The experimental results demonstrate that the method is faster and takes less time to detect in music notation detection. To ensure the wholeness of music notation in note separation, the literature [23] proposed a method to reshape music notation using hidden Markov models and achieved good results in experiments. The researchers in the literature [24] transferred the method to the handwritten data of music notation based on the former and proposed a fusion algorithm of neural network and discriminative algorithm [25], which was able to identify the handwritten data completely and accurately under the ideal situation of unstructured environmental factors.

Among the methods of music notation recognition, most researchers prefer the end-to-end neural network method because the music notation needs to do note segmentation process during the preprocessing process, due to the variability problem of manuscript notes. In the process of note image acquisition, poor image quality, note overlap, note occlusion, and other problems can affect the integrity of note segmentation work. To solve this problem, researchers have used end-to-end neural network recognition methods to extract local and overall note features to ensure the integrity of local features and correct recognition of damaged notes [26, 27]. In addition, researchers in the literature [28, 29] proposed a deep neural network-based note synthesis method for the problem of damaged notes that cannot be correctly recognized, which is mainly based on the local features of notes and automatically improves the defective notes against the note learning library, which has a high dependency on the note learning library. In other words, the richness of the note learning library determines the note recognition accuracy of the method.

## 3. Method

### 3.1. Basic Pipeline

To ensure the feature integrity of the musical score, a generative adversarial network is chosen as the basis for learning from note local features through an unsupervised training mode, which can perform undifferentiated feature reorganization for various images with the aid of computer vision techniques. The generative adversarial network consists of two parts, a generator and a discriminator, which are used to simulate the note features to be learned and generate pseudo-samples with high feature similarity to match them. In the data input stage, only the real note samples that have been preprocessed are segmented, and then the generator simulates similar pseudo-samples based on the feature analysis. The discriminator will score the similarity between the fake samples and the real samples, and the fake samples that meet the specified scoring range will be output directly through the simulator, while the fake samples that do not meet the scoring range will be fed back to the front end to regenerate the fake samples until the fake samples that meet the scoring criteria are generated. The structure of the generative adversarial network is shown in Figure 2.

Generative adversarial networks are based around mutual game learning methods as mathematical principles and are effective in obtaining independent note features in music notation recognition work. For note separation of pentatonic and characteristic scores, the generative adversarial network will optimize the feature editing of the characteristic notes using a pseudo-sample generation model to control the sample output of the note features by editing between discriminator parameters. Such an approach can indirectly control the local and overall features from the notes, avoiding the problem of feature loss in feature separation.

### 3.2. Generator

The generator is a combination of a fully connected neural network and a deconvolutional network. The generator can automatically obtain the key features of the input notes and spectral data based on them and generate pseudo-samples with similar features at the terminals. The principle of generator action is shown in Figure 3. For the pseudo-sample output by the generator, we will discriminate the feature parameters from different dimensions and feedback to the training layer to adjust the feature dimension parameters to get better quality pseudo-samples.

Researchers in the literature [30, 31] aimed to implement the embedded matching problem in feature encoding and decoding. They designed feature encoders with similar specifications at the input and consistent feature decoders at the output, and experimentally demonstrated that such a matching design improved the efficiency of pseudo-sample generation in generative adversarial networks, reduced the number of parameters, and improved the robustness of the networks. Therefore, we also adopt the same combination of decoding and encoding embedded matching, and to make the note feature encoding more adaptable to the embedded model, we also adopt the cascade structure as the network skeleton connection. The input of the encoder is an independent downsampled convolutional layer that can retain the expressed intensity features of the input note features, assuming that the retained features are *I*^low^. After downsampling, the note features will be converted to the hidden layer as a backup. The literature [32] refers to the residual network in the structure design of the decoder, which avoids the problem of note feature information omission during the decoding training process and makes the whole decoding network more compact. We also adopt the same decoder design strategy, and we introduce different levels of residual blocks in the decoder to ensure that note features of different strengths can be fully decoded. In addition to the introduction of residual blocks, the decoder uses the upsampling deconvolutional layer as the main network to realize the conversion between the prescribed expression ranges of note features of different intensities. The convolutional layers in the decoder and encoder uniformly employ normalization operations and ReLU linear activation with a step size of 2. We used the *X* conv operator mentioned in the literature [33], assuming that the given *K* input is (*p*_1_, *p*_2_,…, *p*_*k*_) and the *K* input is the result of a multi-layer perceptron weighting. Then, the *K* × *K* transform matrix Χ=MLP(*p*_1_, *p*_2_,…, *p*_*K*_) is executed and the convolution summation gives the transformed features of the convolution operator X. To solve the adjacency effect between different note features, we have the following mathematical definition for the *X* conv operator.

(1) $$\begin{array}{c} F_{p}=\mathrm{Χ\_}\text{conv}\left(K,p,P,F\right),\\ \mathrm{Χ\_}\text{Conv}\left(K,p,P,F\right)=\text{Conv}\left(K,\text{MLP}\left(P-p\right)\times \left[{\text{MLP}}_{\delta }\left(P-p\right),F\right]\right), \end{array}$$

where *p* denotes the note feature points, *K* denotes the adaptive convolution kernel, *P*=(*p*_1_, *p*_2_,…,*p*_*k*_)^*T*^ denotes the *K* points in its neighborhood, and *F*=(*f*_1_, *f*_2_,…, *f*_*K*_) denotes the features of different notes. Using the principle of Χ conv operator, we construct a musical short note generator representing different intensity features, as shown in Table 1. We replace the connection of the encoder and decoder and use a jump connection structure to ensure that the location information of the random note features matches each other.

### 3.3. Discriminator

The discriminator is the same as the generator and has the same deconvolution network hierarchy. The discriminator evaluates the pseudo-sample output by the generator by using the feature parameters of the real samples as the discriminant criteria. If the evaluation result is not up to the standard, the pseudo-sample is fed back to the generator and the pseudo-sample is generated again. The discriminator is capable of adjusting the parameters according to the note characteristics on its own or manually on demand. The working principle of the discriminator is shown in Figure 4.

The conversion between low-order note features and high-order note features is prone to pitch confusion, and we filter the high-order note features in the generator, compensate the high-order note features by the underlying data density, and distinguish the similarity between high-order and low-order note features by the high-density note feature layer in the discriminator. Researchers in the literature [34] proposed an alternating training model on the problem of optimizing note feature discretization and replaced the mathematical computation in principle with the iteration of maximum and minimum values. We have adopted the same approach, and we have the following mathematical definition for the maximum and minimum value turnover in the evaluation of high- and low-order note features.

(2) $$\begin{array}{c} \frac{\text{min}}{\text{Gen}}\frac{\text{max}}{\text{Dis}}={Ε}_{I}^{\text{high}}\text{log}\left(\text{Dis}\left(I^{\text{high}}\right)\right)+{Ε}_{I}^{\text{low}}\text{log}\left(1-\text{Dis}\left(\text{Gen}\left(I^{\text{low}}\right)\right)\right), \end{array}$$

where Gen denotes the note features generated by the generator and Dis denotes the note features determined by the discriminator. {*I*^low^, *I*^high^} denotes a pair of musical notations with different feature strengths but the same note order. The adversarial loss function equations for generator Gen and discriminator Dis are shown below.

(3) $$\begin{array}{c} L_{G\_\text{adv}}=-\frac{1}{N}\sum_{n=1}^{N}\text{log}\left(\text{Dis}\left(\text{Gen}\left(I_{n}^{\text{low}}\right)\right)\right),\\ L_{D\_\text{adv}}=-\frac{1}{N}\sum_{n=1}^{N}\left\{\text{log}\left(\text{Dis}\left(I_{n}^{\text{high}}\right)\right)+\text{log}\left(1-\text{Dis}\left(\text{Gen}\left(I_{n}^{\text{low}}\right)\right)\right)\right\}, \end{array}$$

where *N* denotes the total number of training note samples. In the process of adversarial neural network convergence, different discriminator parameters are set according to different note strata, and hierarchical restriction means are adopted for pseudo-sample convergence to screen high-order notes and feedback to the generator to generate high-density note features. For this purpose, we established discriminator network layers with different hierarchical structures, and the network layer density information is shown in Table 2.

### 3.4. Loss Function

There is a clear problem of differential differentiation between high-order and low-order notes in the hierarchical feature representation, and the real note feature *I*^high^, modulated by the high-intensity density parameter, guides the generator to synthesize pseudo-samples with highly similar intensity of feature Gen(*I*^low^). The literature [35] mentions a point-by-point loss optimization approach in the pseudo-sample optimization strategy, which constrains the loss function by controlling the relative distance between high-intensity features and low-intensity features. In this paper, we control the feature distance between high-intensity and low-intensity features, constrain the features using the L1 loss function, and increase the integration of features of different classes using the L2 loss function. Our loss function constraint equation is shown below.

(4) $$\begin{array}{c} L_{\text{note}}=\frac{1}{N_{\text{note}}}\sum_{i=1}^{N_{\text{note}}}\left\|\text{Gen}{\left(I^{\text{low}}\right)}_{i}-I_{i}^{\text{high}}\right\|, \end{array}$$

where *N*_note_ denotes the note features in the low-order samples and also denotes the tone spectrum data points in the high-order samples. Combining the above loss functions, the systematic loss function formula of our optimized generative adversarial network is as follows.

(5) $$\begin{array}{c} L=\omega_{1}L_{G\_\text{adv}}+\omega_{2}L_{\text{note}}, \end{array}$$

where *ω*_1_ denotes the weighting coefficient. We adopt the alternating training network iteration mode, and the generator-side network can generate pseudo-samples with very high feature similarity in iterations, which can reduce the discriminator parameter adjustment step when discriminating with the real samples.

### 3.5. Music Notation Recognition Network

For applying a deep neural network model to the recognition of short scores for music teaching, we compared several neural networks in the selection of the underlying network and finally chose a generative adversarial network. The most unique advantage of the generative adversarial network is that it does not affect the original note feature structure, which is regenerated by a generator simulating real samples. We propose an improved generative adversarial network method based on this network to improve the recognition accuracy and recognition speed of music notation. In our improved strategy, the generator and discriminator are embedded together in the residual structure, which can successfully resolve the recognition differences between notes with different data densities. For low-order note data, the convolutional neural network can generate auxiliary samples by downsampling. For high-order note data, the inverse convolutional network upsampling can get the note feature intensity, and then the pseudo-samples can be generated by the feature calculation through the *X* conv operator. In the joint output, different layers of music notation are modeled and filtered with features in the form of note features, and the classifier obtains key features from real samples to provide guidelines for pseudo-sample generation, fusing comprehensive note features. The detailed music notation recognition network is shown in Figure 5.

## 4. Experiment

### 4.1. Datasets

To validate our method for music notation score recognition, we chose a public dataset for experimental validation. The dataset of the music notation series contains 4 categories, which are a monophonic spectrum, polyphonic spectrum, polyphonic spectrum, and mixed spectrum. The most representative dataset in the monophonic category is the Bach Chorales (BC) dataset [36], which is in XML format for the whole series and contains four vocal parts and multiple melodic parts. This dataset has an important role in the melodic generation and harmonic modeling studies. The most famous dataset for polyphonic spectra is the MAESTRO (MO) dataset [37], which is a collection of MIDI-enabled piano melodies, each corresponding to a different audio spectrum, and on which many of Google's spectral studies have been conducted. The most representative dataset for polyphonic scores is the Video Game (VG) dataset [38], where most of the scores are derived from video game music and are mainly used for electroacoustic synthesis. The most famous dataset for mixed scores is the Lakh (LH) dataset [39], which has the advantage of a large number and is mostly used for model pretraining. Besides, we added a wild dataset the Largest MIDI (LM) dataset [40] to ensure the diversity of music notation and to improve the generalization of the music notation recognition model. Details are dataset information as shown in Table 3.

### 4.2. Analysis of Results

To verify the effectiveness of our method for note recognition in music notation, we compared machine learning methods and deep learning methods. Among the machine learning methods, we chose the most representative logistic regression (LR) and decision tree (DT), and among the deep learning algorithms, we chose recurrent neural network (RNN) and long short-term memory network (LSTM). To ensure independent validation relationships between each method, we conducted five sets of experiments during the training process to independently verify the efficiency of each group of methods for sound spectrum recognition. We use recognition accuracy (P), F1 score, and recall rate (*R*) as the evaluation criteria of the music short score recognition methods. Each method detection result will be directly fed into the statistical calculation part of the dataset, and the final evaluation result will be obtained by the balance between the total number and quality of the dataset. To verify the preference of each method in different source datasets, we divided the dataset into two groups. The first group is composed of monophonic scores, polyphonic scores, and polyphonic scores, and this dataset is mainly used to verify the efficiency of the music notation recognition methods for independent recognition of monophonic and polyphonic notes. The experimental results are shown in Table 4.

From the experimental results in the above table, it can be seen that the machine learning method does not perform well enough in the independent recognition experiments for both monophonic and polyphonic spectra, and the accuracy is below 70%. The deep learning method maintains the recognition accuracy between 70% and 86% in the spectrum recognition experiments, and our method achieves an average recognition accuracy of 90% in the spectrum recognition. The experimental results demonstrate that our method has the best independent recognition in both monophonic and polyphonic phonetic spectra. In the second experimental dataset, we chose mixed and wild tone spectra as the base dataset, and this set of experiments is mainly to verify the recognition effect of the tone spectral recognition method in the miscellaneous tone spectra. The experimental results are shown in Table 5.

From the experimental results in the table above, it can be seen that the machine learning method is less efficient in the recognition of the murmur spectrum than the monophonic and polyphonic spectra, and the deep learning method performs generally in the experimental results of the murmur spectrum, with the overall average recognition accuracy remaining at 78%, while our method performs even better in the recognition of the murmur spectrum, with the overall recognition accuracy remaining above 90%. Since our method adopts the separated feature twin method, which does not affect the original note features, it is more efficient in the process of murmur note feature extraction and has higher recognition accuracy. The combined results of all experiments show that our method is better compared to both machine learning methods and deep learning methods.

To verify whether the note information of music notation is accurately recognized, we selected four metrics from the note level: note meta information (NMI), note nodal line (NNL), note chord (NC), and note segmentation (NS). In order not to let the difference in datasets affect the efficiency of note recognition for each method, we selected a common dataset from the monophonic group and the murmuring group for validation, respectively. After the previous experiments, we found that there are significant differences between machine learning methods and deep learning methods. To save experimental costs, this session of experiments will only validate the note recognition efficiency of deep learning methods. The experimental results are shown in Table 6.

The experimental results in the above table show that the overall recognition rate of note details of monophonic notes is higher than that of the miscellaneous note spectrum. The reason for this result is that the monophonic score is more standardized in the segmentation of note detail information, while the miscellaneous score is a mixed scale, which is not standardized in the segmentation, causing the problem of low recognition efficiency. This problem can be adjusted during data preprocessing. Referring to different methods is note recognition efficiency, our method note detail information recognition efficiency is kept above 80%, and our method is significantly better than other deep learning methods.

## 5. Conclusion

Music teaching is often difficult to grasp the characteristics of the notes and tones of the musical notation, and traditional teaching methods do not allow students to have a comprehensive understanding of the notation. This reduces the efficiency of music teaching. To improve the quality and efficiency of music teaching, we try to automate the teaching of music notation. With the addition of computer vision technology and note recognition algorithms, we improve the generative adversarial network to enhance the recognition accuracy and efficiency of music short scores. We adopt an embedded matching structure based on adversarial neural networks, starting from generators and discriminators, respectively, to unify generators and discriminators from the note input side. Each network layer is then laid out according to a cascade structure to preserve the different layers of note features in each convolutional layer. Residual blocks are then inserted in some network layers to break the symmetry of the network structure and enhance the ability of the adversarial network to acquire note features. To validate the efficiency of our method, we selected the monophonic spectral dataset Bach Chorales, the polyphonic spectral dataset Video Game, and the miscellaneous spectral dataset Lakh for validation. The experimental results prove that our method has the best recognition accuracy in both monophonic and miscellaneous phonetic spectra, and in the recognition efficiency of note detail information, our method maintains more than 80%, which is better than other deep learning methods.

Compared with machine learning methods and deep learning methods, our method still has much room for improvement in recognition accuracy and recognition efficiency, although it performs best in the music notation recognition experiments. In future research, we will try to add recurrent neural networks as auxiliary classification in the adversarial network to optimize the recognition of mixed notes during note segmentation and improve the robustness and generalization of the network.

## Figures and Tables

**Figure 1:** Music notation recognition process.

**Figure 2:** Generative adversarial network architecture.

**Figure 3:** Music notation generator process.

**Figure 4:** Music notation discriminator process.

**Figure 5:** Music notation recognition network.

**Table 1:** Detailed hierarchy of generators.

Layer	Type	Detail
1	Input	5001 × 3
2	X conv	Np = 2400, *C* = 16, *K* = 8, *D* = 1
3	X conv	Np = 800, *C* = 64, *K* = 16, *D* = 2
4	X conv	Np = 200, *C* = 256, *K* = 24, *D* = 2
5	X conv	Np = 800, *C* = 64, *K* = 24, *D* = 2
6	X conv	Np = 2400, *C* = 16, *K* = 16, *D* = 2
7	X conv	Np = 5001, *C* = 16, *K* = 16, *D* = 1
8	Fully connected	*C* = 3
9	Output	5001 × 3

**Table 2:** Detailed hierarchy of discriminator.

Layer	Type	Detail
1	Input	5001 × 3
2	X conv	Np = 2400, *C* = 16, *K* = 8, *D* = 1
3	X conv	Np = 800, *C* = 64, *K* = 16, *D* = 2
4	X conv	Np = 200, *C* = 256, *K* = 24, *D* = 2
5	Fully connected	*C* = 1
6	Mean	—
7	Output	1 × 1

**Table 3:** Dataset information.

	Datasets				
	BC	MO	VG	LH	LM
Train	79801	56342	46351	87500	65492
Test	21420	15993	20365	30021	29564
Total	101221	72335	66716	117521	95056

**Table 4:** Comparison of single-tone and multi-tone spectra.

	BC			MO			VG		
	*P*	R	F1	*P*	R	F1	*P*	R	F1
LR	0.57	0.58	0.64	0.63	0.67	0.64	0.63	0.58	0.61
DT	0.69	0.70	0.69	0.70	0.61	0.64	0.68	0.64	0.64
RNN	0.75	0.81	0.82	0.76	0.70	0.71	0.84	0.81	0.77
LSTM	0.81	0.85	0.84	0.81	0.79	0.81	0.86	0.83	0.83
Ours	0.92	0.93	0.88	0.88	0.89	0.87	0.91	0.93	0.91

**Table 5:** Comparison of the recognition effect of the miscellaneous sound spectrum.

	LH			LM		
	*P*	R	F1	*P*	R	F1
LR	0.51	0.53	0.61	0.62	0.53	0.54
DT	0.60	0.63	0.64	0.69	0.62	0.59
RNN	0.71	0.80	0.81	0.77	0.75	0.73
LSTM	0.79	0.83	0.84	0.82	0.82	0.75
Ours	0.90	0.95	0.93	0.92	0.90	0.95

**Table 6:** Notation recognition efficiency of different methods.

	NMI		NNL		NC		NS	
	BC	LH	BC	LH	BC	LH	BC	LH
RNN	0.61	0.51	0.71	0.68	0.81	0.75	0.53	0.41
LSTM	0.73	0.64	0.82	0.75	0.85	0.79	0.62	0.49
Ours	0.86	0.80	0.91	0.89	0.93	0.89	0.81	0.80

## Data Availability

The dataset can be accessed upon request.
